# MiR-98 Protects Nucleus Pulposus Cells against Apoptosis by Targeting TRAIL in Cervical Intervertebral Disc Degeneration

**DOI:** 10.1155/2022/6187272

**Published:** 2022-01-25

**Authors:** Shimin Xu, Yuezhong Li, Junshan Zhang, Zhiwei Li, Yanping Xing

**Affiliations:** Department of Spine Surgery, Weifang People's Hospital, No. 151, Guangwen Street, Kuiwen District, Weifang City, Shandong 261041, China

## Abstract

The excessive apoptosis of nucleus pulposus (NP) cells is a major risk factor in the progress of cervical intervertebral disc degeneration (IVDD). In this study, we investigated the impact of miR-98 on apoptosis of NP cells and the potential molecular mechanisms. Lipopolysaccharide (LPS) was used to establish an NP cell IVDD model. The sponging effect of miR-98 on TRAIL 3′UTR was predicted by ENCORI and assessed by the dual-luciferase reporter gene system. The expression levels of miR-98, TRAIL, and TRAIL pathway-related genes were tested by qRT-PCR, Western blot, and immunofluorescence analysis. Cell apoptosis was analyzed by Hoechst 33258 staining and flow cytometry. Cell viability was analyzed by MTT assay. It was found that the expression level of miR-98 was downregulated, while the level of TRAIL was upregulated in IVDD tissues, and their levels were negatively and positively associated with the clinical MRI grade, respectively. The LPS treatment resulted in a significant decrease of the miR-98 expression level and an increase of the TRAIL expression level in NP cells. miR-98 reduced NP cell apoptosis under LPS treatment in vitro. miR-98 directly targeted TRAIL. Moreover, the mRNA and protein levels of DR5, FADD, cleaved caspase8, cleaved caspase3, and cleaved PARP were downregulated by miR-98 overexpression. Overexpression of TRAIL partially reversed the suppressive roles of miR-98 on cell apoptosis and activation of the TRAIL pathway. We concluded that miR-98 inhibited apoptosis of NP cells by inactivating the TRAIL pathway via targeting TRAIL in IVDD NP cells. These results indicated that miR-98 might be a therapeutic target for IVDD.

## 1. Introduction

Cervical intervertebral disc degeneration (IVDD) is a common clinical disease, and it affects more than 62% of patients whose age was over 40 years, with or without any clinical symptom [1]. IVDD is a causative factor of cervical spondylosis, leading to upper limb numbness, neck or back pain, and dizziness [2]. Many patients with late-stage or severe IVDD will develop cervical spinal stenosis and herniated disc, requiring surgical intervention and causing greater financial burden [2, 3]. Various risk factors affect IVDD including genetic predisposition, mechanical stress, aging, chemical stimulation, and so on [4]. More and more studies indicated that the excessive apoptosis of nucleus pulposus (NP) cells had a vital influence on the progress of IVDD [5]. Thus, it is an important strategy to block the apoptotic pathway and suppress the apoptosis of NP cells for the prevention and treatment of IVDD.

As the small, single-stranded RNAs, microRNAs (miRNAs) could suppress gene expression at the posttranscriptional regulation process or induce target gene mRNA degradation [6]. miRNAs have a vital regulatory role in differentiation, apoptosis, proliferation, carcinogenesis, and drug resistance [7, 8]. Remarkably, accumulating evidence indicates that the levels of miRNAs are frequently dysregulated in intervertebral disc degeneration, which can induce NP cell apoptosis and destroy the balance of cell-matrix synthesis and degradation [7–9], for instance, Sun et al. confirmed that miR-181a directly targeted TRAIL and alleviated the disarrangement of intervertebral disc tissue in intervertebral disc degeneration mice [7]; miR-133a was demonstrated to significantly promote type II collagen expression by targeting MMP9 in NP cells [8]. It has also been found that the expression of miR-98 was dropped in IVDD tissues [9]. It was also reported that the dysregulated miR-98 could decrease type II collagen level, leading to intervertebral disc degeneration through blocking the IL-6/STAT3 signaling pathway [9]. It has also been confirmed that miR-98 prevented the unrestricted expansion of diabetogenic cytotoxic T cells by directly targeting TRAIL and Fas and blocking the apoptosis signaling pathways [10]. So, we hypothesized that miR-98 could have some potential protective effects via inhibiting the NP cell apoptosis in IVDD.

As the common apoptosis-inducing factor, TRAIL is expressed in various tissues and organs (including intervertebral disc tissues), and it can induce apoptosis of cells via binding to TRAIL-specific receptors [11]. In humans, TRAIL interacts with DR4 and DR5 to transduce apoptosis signals [12]. Then, adapter molecules such as Fas-associated death domain (FADD) as well as signaling molecules such as caspase8 were recruited to forming a death-inducing signaling complex (DISC), which is initiated by oligomerization of TRAIL receptors. The DISC induces the proximity and cleavage of caspase8 [13, 14]. Once being activated, the cell death signal is transmitted to downstream events by cleaved caspase8. Caspase3 is one of the substream proteins, which in turn cleaves PARP, thereby culminating in the cell apoptosis [15]. It has been reported that cell apoptosis could be regulated by interfering with the TRAIL-signaling pathway. For example, the overexpression of miR-133a promoted TRAIL resistance by targeting DR5 and blocking the TRAIL-signaling pathway in glioblastoma [16]. Besides, miR-25 targeted DR4 and inhibited TRAIL-induced cholangiocarcinoma apoptosis [12]. The expression levels of TRAIL, DR4, and DR5 are increased in intervertebral disk degeneration cells, which are positively correlated to the degenerative state of the disk [12]. Therefore, it may be a key potential application in the treatment of IVDD by targeting TRAIL and blocking the TRAIL-signaling pathway.

LPS (>1–300 ng/mL) is one of the major components of the Gram-negative bacterial cell wall and is often used as a strong promoter of inflammation, binds to TLR4, leading to the activation of the toll-like receptor signaling pathway [17], which can promote the production of TRAIL [18]. Thus, we established the IVDD model using NP cells treated with LPS. In the current study, we aimed to explore whether miR-98 could target TRAIL in NP cells and assessed the inhibitory impact of miR-98 on NP cell apoptosis stimulated by LPS.

## 2. Materials and Methods

### 2.1. Human NP Tissue Samples

The methodology of the study was approved by the Research Ethics Committee of Weifang People's Hospital (Weifang, China). To obtain human NP tissue at surgery, we got the written consent form from all subjects or their relatives. There were 20 IVDD patients (IVDD; average age 45 ± 1.53; male = 9, female = 11) who underwent spinal fusion or disc resection surgery to relieve neck or back pain and 20 non-IVDD patients (normal; average age 29 ± 2.15; male = 12, female = 8) who underwent traumatic cervical spine fracture participated in our study. All the patients underwent routine MRI scans of the cervical spine before the surgery; then, the degree of cervical disc degeneration was assessed by a modified Pfirrmann classification according to the T2-weighted images [19]. Then, all NP tissue samples were regrouped based on the MRI score and stored in liquid nitrogen at −80°C.

### 2.2. Cells and Cell Culture

ScienCell Research Laboratories (USA) provided human NP cells. The cells were maintained in DMEM (Gibco, USA) supplementing with 10% FBS (Gibco, USA) and 1% antibiotics. The NP cells were treated with 0.01–10 *μ*g/mL of LPS (Sigma-Aldrich, USA) for 12–48 h to trigger cell inflammation in vitro.

### 2.3. Cell Transfection

MiR-98 mimics and its control (mimics-NC) were purchased from Applied Biosystems (USA). TRAIL pcDNA 3.1 (pcDNA-TRAIL) was designed and synthesized by GenePharma (China). Lipofectamine 2000 (Thermo Fisher, USA) was used to transfect the miRNAs and pcDNA-TRAIL into NP cells. After 24 h of transfection, 1 *μ*g/mL LPS (Sigma-Aldrich, USA) was applied to stimulate the cells in DMEM (Gibco, USA). We collected the cells after 24 h for subsequent experimentation.

### 2.4. Real-Time Quantitative PCR

To extract RNA from the samples, TRIzol reagent (Thermo Fisher, USA) was used. For small RNA (smaller than 200 nucleotides in size), the mirVana miRNA isolation kit (Austin, USA) was used to isolate small RNA from total RNA. For mRNA, RNA was reversely transcribed into complementary DNA (cDNA) with a reverse transcription cDNA kit (Thermo Fisher, USA). qRT-PCR was conducted via the SYBR-Green PCR SuperMix-UDG kit (Thermo Fisher, USA) under the Opticon RT-PCR Detection System (ABI 7500; Thermo Fisher, USA). For miRNA, the TaqMan microRNA Reverse Transcription Kit (Thermo Fisher, USA) was selected to perform RT reactions. Subsequently, conventional TaqMan PCR (Thermo Fisher, USA) was used to quantify the RT product. U6 and GAPDH were used for normalization.  Table 1 provides all the sequences of primers, which were purchased from GenePharma (China). The 2^−ΔΔCt^ method was used to calculate the relative expression [20].

### 2.5. Western Blot

After extracted total protein from NP cells and NP tissues with RIPA buffer (Cell Signaling Technology, USA), the samples were transferred into a polyvinylidene fluoride membrane (PVDF, Millipore), and electrophoresis was conducted to separate the samples with a 10% SDS-PAGE gel (Solarbio, China). The protein concentration was quantified by a BCA assay kit (Sigma-Aldrich; USA). The primary antibodies were TRAIL (Rabbit; 3219; 1 : 1000), DR5 (Rabbit; 8074; 1 : 1000), FADD (Rabbit; 2782; 1 : 1000), caspase8 (Mouse; 9746; 1 : 1000), cleaved caspase8 (Rabbit; 8592; 1 : 1000), caspase3 (Rabbit; 9662; 1 : 1000), cleaved caspase3 (Rabbit; 9661; 1 : 1000), PARP (Rabbit; 9532; 1 : 1000), cleaved PRAP (Rabbit; 5625; 1 : 1000), and GAPDH (Rabbit; 5174; 1 : 1000) specific. All antibodies were bought from Cell Signaling Technology, the USA. Then, we added the secondary antibodies (goat anti-mouse/rabbit IgG; Abcam, UK), which were conjugated with horseradish peroxidase (HRP) (CST, USA). ImageJ software (version 5.0; Bio-Rad, the USA) was applied to analyze and quantify the gray value of the strips. GAPDH was used as a control.

### 2.6. MTT Assay

The cytotoxic assay was detected using an MTT kit (Solarbio, China). The transfected cells were seeded in a 96-well plate in 200 *μ*l medium. At the specified point in time, 100 *μ*l culture medium containing 20 *μ*l MTT was added into each well, and then, the 96-well plates were placed in the incubator. After 4 h, 150 ul/well formazan solution was used to dissolve the blue-purple crystals. The optical density value was read using a microplate reader (Thermo Fisher, USA) at 490 nm.

### 2.7. Hoechst 33258 Staining

Sterile glass coverslips with 24-well plates were used for cell seeding, and every well had 5 × 10^4^ cells. After different treatments, the cells were isolated from the medium, fixed using 4% paraformaldehyde (Solarbio, China) for 15 min, washed using 0.15 mol/L NaCl for 3 times, and stained using 2 *μ*g/mL Hoechst 33258 (Sigma-Aldrich; USA) in HBSS for 5 min. After washing with 0.15 mol/L NaCl for 2 times, the antifade mounting medium (Beyotime, China) was used to mount the coverslips onto slides. The fluorescence microscope (Olympus IX50, Japan) was used to observe the morphologic changes in apoptotic nuclei.

### 2.8. Flow Cytometry Analysis

Annexin V-FITC-propidium iodide (PI) apoptosis detection reagent (BD Biosciences, USA) was selected to test cell apoptosis as previously described [21]. Briefly, PBS was used to wash the NP cells 3 times, and the NP cells were digested with trypsin (1 mL) and resuspended using 1X Annexin binding buffer at 1 × 10^5^ cells/100 *μ*l. Then, we gathered and stained the cells with Annexin V-FITC and PI for 15 min. Finally, flow cytometry (version 10.0, FlowJo, FACS Calibur^TM^, BD Biosciences, USA) was used to count the cells.

### 2.9. Dual-Luciferase Reporter Assay

The putative binding sites of miR-98 in 3′-UTR of TRAIL was predicted by ENCORI. The pMIR-reporter plasmids (Huayueyang, China) named TRAIL-WT and TRAIL-MUT with wild-type and mutated 3′-UTR of TRAIL mRNA were constructed. Briefly, the mutation site of the binding region of miR-98 in 3′-UTR TRAIL was designed. The cDNA fragments of TRAIL (3′-UTR) containing the wild-type (WT) or mutant-type (MUT) were amplified. Restriction enzyme sites SpeI and Hind III were used to introduce the cDNA fragments into pMIR-reporter. The sequenced luciferase MUT and WT reporter plasmids were, respectively, cotransfected with miR-98 into NP cells. To determine the luciferase activity, the dual-luciferase reporter assay system (Promega, USA) was applied 30 h after transfection. Renilla luciferase activity was used to normalize the results.

### 2.10. Immunofluorescent Assay

The NP cells were first fixed in 4% paraformaldehyde and incubated overnight in primary rabbit polyclonal anti-TRAIL, polyclonal rabbit anti-DR5, or anticleaved caspase8 (CST, the USA) antibodies, respectively. On the next day, the cells were treated with the Alexa Fluor®594 labeled conjugated goat-rabbit IgG, and cell nuclei were counterstained with DAPI (Beyotime, China). The results were observed under an Olympus FluoView 2000 laser scanning confocal microscope (Olympus, Japan).

### 2.11. Statistical Analysis

Statistical analysis was carried out using Prism 8 (GraphPad Software, the USA). To evaluate statistically significant differences between two groups, one-way ANOVA or Student's *t*-test was performed. The chi-square test was used for the comparative analysis of the discontinuous variables (Table 2). The statistically significant differences were indicated by *P* < 0.05.

## 3. Results

### 3.1. The High Expression of TRAIL and Low Expression of miR-98 in IVDD Tissues

The expressions of TRAIL and miR-98 and the clinical characteristics of the patients with IVDD were assessed and are given in Table 2. A high TRAIL expression (higher than mean) was correlated with a high MRI grade, while the correlation between the miR-98 level and MRI grade showed the opposite results. However, the levels of miR-98 and TRAIL were not correlated with age, sex, or body mass index.

The relative expressions of miR-98 and TRAIL were detected by qRT-PCR in NP tissues (normal vs. IVDD, Figures 1(a) and 1(b)). The results showed that the expression of miR-98 was significantly lower in IVDD tissues than in the normal control (*P* < 0.01). In contrast, TRAIL mRNA expression was significantly higher (*P* < 0.01). The representative results of Western blot assay confirmed the results of qRT-PCR (Figure 1(c)). Moreover, it showed a negative correlation between the expression of miR-98 and TRAIL expression (*r* = −0.5977, *P* < 0.05) (Figure 1(d)).

### 3.2. Establishment of the IVDD Cell Model

To find the appropriate concentration and treatment time of LPS, we used different LPS concentrations (0.01–10 *μ*g/mL) and treatment periods (0, 12, 24, and 48 h) to stimulate NP cells and assessed the cytotoxic effect using MTT assay. It was found that the viability of NP cells reduced with the increase of LPS concentration and treatment time duration. As shown in Figure 2(a), the cell viability was significantly decreased with 1 *μ*g/mL (24 h and 48 h) and 10 *μ*g/mL (24 h and 48 h) LPS (*P* < 0.05). However, it dropped below 50% with 1 *μ*g/mL (48 h) and 10 *μ*g/mL (24 h and 48 h) LPS. Then, the expressions of miR-98 and TRAIL in the IVDD cell model treated with LPS were detected. As predicted, qRT-PCR analysis demonstrated that TRAIL expression was upregulated in NP cells stimulated with the increase of LPS concentrations (0.01–1 *μ*g/mL; 24 h), but it dropped under 10 *μ*g/mL LPS treatment (Figure 2(b)), and the results of Western blot assay were consistent with the results of qRT-PCR (Figure 2(c)). The highest level of TRAIL expression was observed under 1 *μ*g/mL LPS (*P* < 0.01 vs. the blank). By contrast, the level of miR-98 was downregulated with the increase of LPS concentrations (Figure 2(d)). Taken together, the IVDD cell model was successfully established with 1 *μ*g/mL LPS treated for 24 h, and miR-98 was significantly downregulated (*P* < 0.01) and TRAIL was significantly upregulated (*P* < 0.01) in response to LPS stimulation in the IVDD cell model.

### 3.3. Overexpression of miR-98 Inhibited LPS-Induced NP Cell Apoptosis

To examine the role of miR-98 in the apoptosis of LPS-induced NP cells, the cells transfected with mimics-NC and miR-98 mimics were divided into 4 groups (blank, LPS, LPS + mimics-NC, and LPS + miR-98 mimics), and high transfection efficiency was verified by qRT-PCR (Figure 3(a)). The results of MTT assay suggested that the cell viability was significantly reduced under the stimulation of LPS in comparison to the blank (*P* < 0.01, Figure 3(b)), while the transfection of miR-98 mimics could significantly increase the cell viability in comparison with the LPS + mimics-NC group (*P* < 0.01, Figure 3(b)). Both flow cytometric analysis and Hoechst 33258 staining were performed, and the results reported that the LPS treatment could significantly increase NP cell apoptosis in comparison to the blank group (*P* < 0.01, Figures 3(c) and 3(d)). In contrast, the transfection of miR-98 mimics significantly decreased NP cell apoptosis in comparison with the LPS + mimics-NC group (*P* < 0.01, Figures 3(c) and 3(d)). These results above revealed that miR-98 could increase cell viability and inhibit apoptosis of LPS-induced NP cells.

### 3.4. MiR-98 Directly Targeted 3′-UTR of TRAIL

To make a further insight into the suppression role of miR-98 on NP cell apoptosis in IVDD, the relationship between TRAIL and miR-98 was investigated. According to the prediction of ENCORI, miR-98 could specifically bind to the 3′-UTR of TRAIL (Figure 4(a)). As shown in Figure 4(b), these predictions were demonstrated by dual-luciferase gene reporter assay in NP cells. The results suggested that the transfection of miR-98 mimics significantly dropped the luciferase activity of the TRAIL-WT group in comparison to the group transfected with mimics-NC (*P* < 0.01). There was no significant difference found between the luciferase activity of the TRAIL-MUT group transfected with miR-98 mimics or mimics-NC (*P* > 0.05). To verify this result, we assessed the level of TRAIL in NP cells transfected with miR-98 mimics and mimics-NC. The results of qRT-PCR reported that TRAIL was significantly lower in the LPS + miR-98 mimics group than in the LPS + mimics-NC group (*P* < 0.01, Figure 4(c)). Western blotting and immunofluorescence assay reported similar outcomes (*P* < 0.01, Figures 4(d) and 4(e)).

### 3.5. MiR-98 Decreased the Apoptosis of NP Cells by Targeting TRAIL

As the transfection of miR-98 mimics repressed the TRAIL levels in NP cells and inhibited apoptosis of NP cells, we then determined whether the transfection of pcDNA-TRAIL could counteract the inhibitory impact of miR-98 on apoptosis of NP cells. The NP cells stimulated with LPS were divided into 5 groups (blank, LPS + pcDNA-NC, LPS + pcDNA-TRAIL, LPS + miR-98 mimics + pcDNA-NC, and LPS + miR-98 mimics + pcDNA-TRAIL). The results of qRT-PCR and Western blot assay showed that pcDNA-TRAIL has been successfully transfected into the NP cells and effectively expressed (Figures 5(a) and 5(b)). We further detected the viability and apoptosis of LPS-treated NP cells, and the results of MTT assays and flow cytometry revealed that miR-98 significantly enhanced the cell viability and suppressed cell apoptosis, and its effects could be effectively reversed by TRAIL (*P* < 0.01; Figures 5(c) and 5(d)).

### 3.6. MiR-98 Targeted TRAIL to Inhibit the Apoptosis of NP Cells via Inactivation of the TRAIL-Signaling Pathway

To assess the roles of miR-98 on the inactivation of the TRAIL-signaling pathway, the NP cells stimulated with LPS were divided into 5 groups as described above. Then, we measured the expressions of DR5, FADD, caspase8, cleaved caspase8, caspase3, cleaved caspase3, PARP, and cleaved PARP by Western blotting (Figure 6(a)). The results demonstrated that the levels of DR5, FADD, cleaved caspase8, cleaved caspase3, and cleaved PARP were significantly increased in the LPS-stimulated group in comparison with the control (*P* < 0.01). Transfection of miR-98 mimics significantly inhibited the pathway by downregulating the expressions of DR5, FADD, cleaved caspase8, cleaved caspase3, and cleaved PARP in LPS + miR-98 mimics + pcDNA-NC in comparison to those in LPS + pcDNA-NC (*P* < 0.01). While, transfection of pcDNA-TRAIL partially reversed the inhibitory of miR-98 mimics and markedly activated this pathway by upregulating their levels in LPS + miR-98 mimics + pcDNA-TRAIL in comparison with that in LPS + miR-98 mimics + pcDNA-NC (*P* < 0.01; Figure 6(a)). The immunofluorescence analysis of DR5 and cleaved caspase8 obtained similar results (Figures 6(b) and 6(c)). These results above showed that LPS activated the TRAIL-signaling pathway, and the suppressive effects of miR-98 on this pathway could be counteracted by TRAIL.

## 4. Discussion

IVDD is a multifactorial disease, but its pathogenesis is still not completely cleared. Degradation of the extracellular matrix, cell loss (apoptosis), and inflammation are all the prevalent pathological changes in IVDD, which are associated with disc degeneration [22]. According to the understanding of IVDD and current knowledge, there are several limitations in standard therapy, such as modest success rates, invasiveness, and high costs [23]. It has been reported that miRNAs were being the most promising approach for IVDD [24]. Particular attention has been paid to the expression of miRNAs and their functions in relieving the symptoms of IVDD. The studies conducted in vivo experiments using the IVDD rat model identified that miR-185 and miR-143-5p were connected with NP cell apoptosis in IVDD [25, 26]. miR-98 could reduce apoptosis in many diseases, such as sepsis and acute myocardial infarction [27, 28]. Nevertheless, the roles of miR-98 in NP cell apoptosis has not yet been studied. In the current study, we discovered that the miR-98 level was lower in IVDD tissues, while the level of TRAIL was significantly higher, and both of them were associated with the grade of disc degeneration. Ji et al.' study also reported similar results [9]. In addition, we also found that there was a negative relationship between the expression of miR-98 and TRAIL levels. NP cell apoptosis played a key role in IVDD, which is mainly induced by TRAIL [12]. To explore the inhibition of miR-98 on apoptosis of NP cells in IVDD, we studied the association between TRAIL and miR-98 in NP cells.

LPS, as a potent inducer of inflammation, can bind to TLR4 and induce cell apoptosis by promoting the production of TRAIL [29, 30]. Thus, in the current study, LPS was used to establish the IVDD cell model for research; then, we obtained the results that the expression of miR-98 was dropped in human NP cells by LPS stimulation, while TRAIL expressions were raised. These results were similar to the previous studies which indicated that the miR-98 level was significantly decreased following LPS stimulation [31, 32], while LPS could increase the expression of TRAIL [30, 33, 34]. In the present study, compared with the stimulation with LPS only, cell apoptosis was suppressed by the overexpression of miR-98. Our study proved that miR-98 played a key role in IVDD partially by inhibiting NP cell apoptosis. These results accorded closely with the previous study of Ji et al. [9].

The putative binding region of miR-98 in 3′-UTR TRAIL was mutated, and a dual-luciferase gene reporter assay demonstrated that miR-98 targeted TRAIL directly; this result was consistent with the previous study of Jong et al. [10]. We also observed that TRAIL expression was significantly reduced following transfection of miR-98 mimics. Besides, to better explore the role of TRAIL in IVDD, pcDNA-TRAIL was transfected into the NP cells, and the results suggested that TRAIL reversed the inhibitory role of miR-98 mimics on the apoptosis of LPS-treated NP cells.

It is well known that the TRAIL-signaling pathway mediates the apoptosis of NP cells in IVDD. DR5, FADD, caspase8, and the downstream caspases are the apoptosis genes involved in the TRAIL-signaling pathway [12, 35]. Previous studies indicated that TRAIL, DR4, DR5, cleaved caspase8, and cleaved PRAP were highly expressed in IVDD cells, and these protein levels were positively correlated with the degenerative state of the disk [12, 35]. Li et al. found that, in contrast with the normal group, there was a highly expressed level of FADD in NP cells of rats in the IVDD model group [36]. Overexpression of miR-98 inhibited the upregulation of DR5, FADD, cleaved caspase8, cleaved caspase3, and cleaved PARP expression induced by LPS. The inhibitory effects of miR-98 mimics on the apoptosis genes expressions could be reversed by the transfection of pcDNA-TRAIL.

## 5. Conclusion

This study found that miR-98 expression was dropped in IVDD and participated in the apoptosis of NP cells by inhibiting TRAIL. More functional model experiments in vivo are needed in the future to verify the effect of miR-98 on IVDD. MiR-98 alleviated IVDD by decreasing the apoptosis of NP cells through inhibiting TRAIL and its downstream apoptosis genes expressions in NP cells. The results provided a deeper opinion into the study of IVDD and suggested that miR-98 might prove to be of regulatory importance of IVDD.

## Figures and Tables

**Figure 1:** TRAIL was highly expressed while miR-98 was low expressed in patients with IVDD. (a) The results of qRT-PCR showed that the miR-98 expression level significantly downregulated in IVDD NP tissues in comparison with normal NP tissues. *P* ≤ 0.001. (b)-(c) The results of qRT-PCR and Western blotting showed that the TRAIL expression level significantly upregulated in IVDD NP tissues compared with normal NP tissues. *P* ≤ 0.001. (d) The correlation between the expression level of TRAIL and miR-98 showing a negative correlation in IVDD NP tissues. ^*∗*^*P* < 0.05 and ^*∗*^*P* < 0.01.

**Figure 2:** Establishment of the IVDD cell model. (a) The NP cells treated with different concentrations and different times of LPS and MTT assay performed to determine the cell viability. (b)–(d) qRT-PCR and Western blotting performed to examine miR-98 and TRAIL expression levels in the NP cells treated by LPS. ^*∗*^*P* < 0.05 and ^*∗*^*P* < 0.01.

**Figure 3:** Overexpression of miR-98 decreased LPS-induced NP cell apoptosis. (a) Transfection efficiency of mimics-NC, miR-98 mimics determined by qRT-PCR. (b) The cell viability of NP cells treated with LPS performed by MTT assay. (c)-(d) NP cell apoptosis after different treatments (blank, LPS, LPS + mimics-NC, and LPS + miR-98 mimics) analyzed by Hoechst 33258 staining and flow cytometry. ^*∗*^*P* < 0.05 and ^*∗*^*P* < 0.01; ^#^*P* < 0.05 and ^##^*P* < 0.01. Scale bars: 50 *μ*m.

**Figure 4:** miR-98 directly targeted 3′-UTR of TRAIL. (a) The 3′UTR of TRAIL predicted as a miR-98 target using ENCORI. (b) Luciferase activity of a reporter containing a wild-type (WT) TRAIL 3′UTR or a mutant (MUT) TRAIL 3′UTR. (c)–(e) The expression level of TRAIL after different treatments (blank, LPS, LPS + mimics-NC, and LPS + miR-98 mimics) determined by qRT-PCR, Western blotting, and immunofluorescence assay. ^*∗*^*P* < 0.05 and ^*∗*^*P* < 0.01. Scale bars: 50 *μ*m.

**Figure 5:** Overexpression of TRAIL reversed the inhibitory effects of miR-98 mimics on NP cell apoptosis stimulated by LPS. (a) Transfection efficiency of pcDNA-NC, pcDNA-TRAIL determined by qRT-PCR. (b) TRAIL protein levels determined by Western blot analysis in different groups (blank, LPS + pcDNA-NC, LPS + pcDNA-TRAIL, LPS + miR-98 mimics + pcDNA-NC, and LPS + miR-98 mimics + pcDNA-TRAIL). (c) The cell viability of NP cells performed by MTT assay in different groups (blank, LPS + pcDNA-NC, LPS + pcDNA-TRAIL, LPS + miR-98 mimics + pcDNA-NC, and LPS + miR-98 mimics + pcDNA-TRAIL). (d) NP cell apoptosis analyzed by flow cytometry in different groups (blank, LPS + pcDNA-NC, LPS + pcDNA-TRAIL, LPS + miR-98 mimics + pcDNA-NC, and LPS + miR-98 mimics + pcDNA-TRAIL). ^*∗*^*P* < 0.05 and ^*∗*^*P* < 0.01; ^#^*P* < 0.05 and ^##^*P* < 0.01; ^@^*P* < 0.05 and ^@@^*P* < 0.01.

**Figure 6:** Overexpression of TRAIL reversed the inhibitory effects of miR-98 on the TRAIL pathway. (a) The protein expression levels of DR5, FADD, cleaved caspase8, caspase8, cleaved caspase3, caspase3, cleaved PARP, and PARP examined by Western blot analysis in different groups (blank, LPS + pcDNA-NC, LPS + pcDNA-TRAIL, LPS + miR-98 mimics + pcDNA-NC, and LPS + miR-98 mimics + pcDNA-TRAIL). (b)-(c). The expression levels of DR5 and cleaved caspase8 also detected by immunofluorescence assay in different groups (blank, LPS + pcDNA-NC, LPS + pcDNA-TRAIL, LPS + miR-98 mimics + pcDNA-NC, and LPS + miR-98 mimics + pcDNA-TRAIL). ^*∗*^*P* < 0.05 and ^*∗*^*P* < 0.01. Scale bars: 50 *μ*m.

**Table 1:** The primer sequences.

Gene	Primer sequence
TRAIL	Forward 5′-GACCTGCGTGCTGATC-3′
	Reverse 5′-TAAAAGAAGATGACAG-3′
miR-98	Forward 5′-UGAGGUAGUAAGUUGUAUUGUU-3′
	Reverse 5′-AACAAUACAACUUCUACCUCA-3′
U6	Forward: 5′-CGCTTCGGCAGCACATATAC-3′
	Reverse: 5′-AAATATGGAACGCTTCACGA-3′
GAPDH	Forward: 5′-GCACCGTCAAGGCTGAGAAC-3′
	Reverse: 5′-TGGTGAAGACGCCAGTGGA-3′

**Table 2:** Association between miR-98/TRAIL expression and the clinical characteristics of patients with IVDD.

Characteristics	miR-98 expression		*P* value	TRAIL expression		*P* value
	Low (12)	High (8)		Low (7)	High (13)	
Ages			0.489			0.158
≤45	4	5		3	6	
>45	8	3		4	7	
Gender			0.145			0.325
Male	7	2		5	4	
Female	5	6		2	9	
Body mass index			0.216			0.173
≤24 kg/m^2^	3	5		1	7	
>24 kg/m^2^	9	3		6	6	
MRI grade			0.028^*∗*^			0.042^*∗*^
G (I/II/III)	2	4		3	3	
G (IV/V)	10	4		4	10	

^*∗*^ *P* < 0.05, statistical significance.

## Data Availability

The data used to support the findings of this study are available from the corresponding author upon request.

## Abbreviations

NP: Nucleus pulposus
IVDD: Intervertebral disc degeneration
LPS: Lipopolysaccharide
MiR: MicroRNA
FADD: Fas-associated death domain
DISC: Death-inducing signaling complex
PCR: Polymerase chain reaction
TRAIL: TNF-related apoptosis-inducing ligand
TLR4: Toll-like receptor 4.
